The article "A Survey of Teachers' Status in Mental Health Education Management Based on Big Data Analysis" was retracted in 2023. Reasons: signs of a paper mill; suspected computer-generated content; unreliable results or conclusions; concerns about the data.

# A Survey of Teachers' Status in Mental Health Education Management Based on Big Data Analysis

**DOI:** 10.1155/2022/8399938

**Published:** 2022-09-21

**Authors:** Yuxi Wang, Chunmei Xue, Minmeng Zhang

**Affiliations:** ^1^School of Modern Languages and Linguistics University of Southampton, Southampton, SO171BJ, UK; ^2^School of Foreign Languages Zhengzhou Sias University, Xinzheng Henan 451100, China; ^3^School of Art Henan University of Finance and Economics, Zhengzhou Henan 450000, China

## Abstract

This paper uses the theory of mental health education to conduct an in-depth study and analysis of teachers' educational management, and based on this, it designs a survey method on teachers' status and analyzes its strategic methods based on the results of the survey. Using literature analysis, questionnaires, survey interviews, and statistical analysis, the analysis of mental health of primary and secondary school teachers in the city was made. The results of the survey and analysis of the questionnaire results were used to construct a compatible mental health evaluation model. It was found that the overall level of elementary school teachers' mental health is poor at present, and different levels of mental health were presented with school sections and ages. A total of 286 questionnaires were distributed, 278 valid questionnaires were returned, and statistical analysis was conducted using EXCEL tables based on the collected data. The data analysis results show that the mental health level of teachers in middle school is significantly lower than that of teachers in primary school, and the mental health level of teachers in primary and secondary schools decreases with the increase of age. Therefore, to prevent the small and the gradual, start from the source; do a good job in the publicity of mental health education in peacetime; popularize the knowledge of mental health, so that teachers have a correct understanding of mental health education; improve the professional level of teachers; set up professional teachers in professional positions; establish sound job system and evaluation system, etc. Promote the balanced development of school psychological counseling rooms, strengthen the construction of professional teachers in mental health education, improve various systems of mental health education, comprehensively popularize teachers' mental health education and training, and mobilize teachers' enthusiasm for scientific research on mental health education. Improve the understanding of mental health education in colleges and universities, and regard mental health education as the foundation of all education.

## 1. Introduction

It is impossible to imagine what kind of changes the growth of the Internet may bring to life in the future, but it is important to admit that we have become completely inseparable from the Internet in our work, study, and life. In this unprecedented new era, we can no longer train students according to the traditional classroom teaching model—teachers speak and students listen [1]. We need to change the traditional concept of education even more. With the rapid development of Internet+ education, the communication and interaction between teachers and students have also changed: previously, it was a single real world, but now, it is reality and virtual parallel. It was offline communication, but now, it is online and offline communication at the same time; previously, teacher-student interaction was mainly in the classroom, but now, it is both classroom and offline interaction through the Internet. Especially in these years, with the rapid development of society, increasingly fierce competition, coupled with the rapid development of industry and commerce, as well as the family planning policy has been implemented; the family structure has changed dramatically; face-to-face communication and interaction between people have been reduced so that the human touch is gradually thin. In people due to the lack of emotional support, which easily causes excessive stress in the work, with the increase in pressure, mental illnesses with times also show a trend of gradually spreading [2]. Teachers are role models for students and are the people who have the most contact with students other than their parents. Teachers have a special status and have the greatest influence on students. Therefore, our middle school teachers must have healthy psychology to cultivate a generation of healthy young people who will realize the Chinese Dream of the great rejuvenation of the Chinese nation. Especially today, with the rapid development of information technology, the Internet has penetrated all aspects of education, and education has encountered unprecedented opportunities and challenges. Our teachers are not spared either. In such a context, we should pay more attention to the occupational stress of junior high school teachers and take favorable measures to prevent and reduce it.

The article "A Survey of Teachers' Status in Mental Health Education Management Based on Big Data Analysis" was retracted in 2023. Reasons: signs of a paper mill; suspected computer-generated content; unreliable results or conclusions; concerns about the data.

The process of selective reception of influence and the interaction between teacher and student allow the achievement of educational goals. The communicative, nontechnical, emotional element between the teacher and the student makes the student a self-developing person. Teachers with a high level of psychological well-being have a strong prosocial behavior, can analyze problems with a rational and calm mind, and improve the students' ability to think and think [3]. Teachers with good professional development have a high level of subjective quality of life, can make students feel positive in their interactions with them, and guide them to love and respect life. Education is the shaping of humanity and the improvement of the quality of life. Teachers love education and have a good state of professional mental health and high quality of survival to take up the responsibility and mission of education. Teachers' psychological problems are, in a sense, a reflection of social problems in teachers, so it is important to create a relaxed and pleasant working and living environment for teachers in every way possible. The comprehensive launch of the “Teachers' Mental Health Education Social Project,” the inclusion of mental health education in teachers' assessment programs and continuing education, and the opening of “teachers' counseling rooms” in primary and secondary schools are important ways to relieve teachers' stress [4]. Education administrators should take the initiative to solve the problems of teachers and try to create a harmonious inner environment for teachers. However, due to its location, it is far from the city center, so there is a big difference in the allocation of educational teachers compared to the more developed areas in the city center. Give full play to the policy-oriented role, tilt to rural schools in title evaluation, cadre selection, merit evaluation, etc. and set up additional rural teacher allowances, rural classroom teacher allowances, and open teacher shuttle buses to mobilize rural teachers to work and attract young teachers to teach in rural areas.

Based on the current situation of colleges and universities and the actual situation of current school students, this paper attempts to further improve the mental health education work in colleges and universities from three levels, including managers, educators, and educated people. Specifically, we create and improve the management system, management mechanism, and evaluation system at the manager level; build and standardize the structure system, operation system, and plan system at the educator level; and refine and deepen the target system, process system, and evaluation system at the educated level [5]. This is also the basic work to carry out the management system of college students' mental health education, which is directly related to the concrete realization of the goal of cultivating qualified talents in colleges and universities. This brings new challenges to the ideological and political education work and moral education work of colleges and universities. This idea has been put forward in various documents and political conferences on strengthening moral education work in schools, and it has been emphasized that one of the important tasks of moral education in colleges and universities is the mental health education of college students, and this task has also been imminent, and the improvement of college students' psychological quality is urgent for their ideological quality [6]. We analyze the outstanding problems of the mental health education management system in general secondary schools from the aspects of education and management and analyze the reasons for them, to provide a theoretical basis for the improvement and promotion of mental health education in secondary schools with good theoretical and Wanfa mental health education system, and prepare for the improvement and promotion of mental health education in secondary schools with theoretical, methodological, and empirical evidence. The mental health of primary and secondary school teachers affects students' learning and growth to a certain extent, which in turn affects the national basic education and even the hope of the country and the nation. Therefore, this paper is aimed at studying the current situation of the mental health level of primary and secondary school teachers in the city, finding out the main factors that affect the mental health of primary and secondary school teachers, and finding limited ways to improve the mental health level of primary and secondary school teachers, relying on the theory of humanism, starting from improving the mental health level of primary and secondary school teachers, designing a questionnaire that can effectively reflect the current situation of primary and secondary school teachers' mental health, constructing an index model for evaluating the mental health of primary and secondary school teachers, and combining actual research data to analyze the causes of middle and primary school teachers. Elementary school teachers have the deficiencies of mental health problems, and according to the empirical results, put forward countermeasures and suggestions to improve the mental health level of primary and middle school teachers.

The article "A Survey of Teachers' Status in Mental Health Education Management Based on Big Data Analysis" was retracted in 2023. Reasons: signs of a paper mill; suspected computer-generated content; unreliable results or conclusions; concerns about the data.

## 2. Related Works

The psychoanalytic doctrine founded by psychologist Sigmund Freud greatly advanced the development of psychotherapy for the world. Shernoff E S is recognized by the American psychological community as the earliest practitioner of mental health education in schools [7]. He began his commitment to mental health education in schools by establishing a relatively complete training system at the University of Pennsylvania, starting with a clinical course dedicated to providing psychological diagnosis and special psychological training for students who were lagging. During this time, the first journal of clinical psychology was founded. School mental health education began to shift its goal to improve students' mental management skills and the development of mental health for prevention. In the United States, the qualifications, induction training, specific functions, and professional norms for school mental health education practitioners were clearly defined and are used to this day, featuring both theoretical and practical work [8]. With the in-depth study of mental health education in schools, psychologists found that it is not enough to focus only on students' psychological development in schools, but it is necessary to include families, teachers, or other people in creating a good mental health education environment for students, to enhance the development of students' psychological abilities and the effectiveness of psychological interventions. As a result, psychologists have begun to work on building a holistic and ecological mental health environment for students. If the first physical protective reaction does not exclude the threat in this area, the stress continues to exist. When the human body must get used to this stress in a certain situation, the secretion of chemical components triggered by physiological reactions in the human body can only be kept at a low level.

In their article, Tang et al. note that when asked about the psychological stress of teachers, 78% of those surveyed would still choose to teach if they had to choose their career again; but when asked the same question again 20 years later, only 46.4% agreed to choose to teach [9]. This is somehow a true reflection of the psychology of teachers; as time goes by, their love for their job is decreasing, while on the contrary, all kinds of dissatisfaction are deepening, and in the same survey, more people feel that the psychological pressure from the profession is threatening the health of teachers. A special survey was conducted in which 300 questionnaires were randomly selected from urban and suburban areas of Beijing, and 93.1% of the teachers found that being a teacher was becoming increasingly difficult and stressful and agreed that this was the main source of anxiety in their work and life. Other scholars have conducted similar surveys since then, and their results also showed that more than 50% of teachers felt more stressed at work [10]. The study by Wang et al. pointed out that the occupational stress and mental health problems of primary and secondary school teachers have reached a time when they have to be paid attention to, which to some extent indicates that Chinese scholars and foreign experts have reached a consensus on the occupational stress of teachers and also indicates that the current teaching profession has become a definitive high-stress profession, and its development trend is becoming more and more serious with the development of economy and society and time [11]. This proves that the phenomenon of occupational stress among primary and secondary school and garden teachers in China must be paid great attention to by the relevant departments.

The article "A Survey of Teachers' Status in Mental Health Education Management Based on Big Data Analysis" was retracted in 2023. Reasons: signs of a paper mill; suspected computer-generated content; unreliable results or conclusions; concerns about the data.

Mental health education was initially explored by some schools on their initiative and then gradually transformed into an official-led promotion with the promulgation of various policies. Although school mental health education in Shanghai started early in the country and the current level of school mental health education management is leading in China, it still faces several problems and shortcomings that need to be further explored and promoted [12]. The organization and implementation of school mental health education are conducive to cultivating positive psychological qualities, improving students' overall quality, and promoting their overall physical and mental development. Strengthening the organization and implementation of mental health education in schools is of great significance for achieving the goal of moral education, promoting quality education for students, and building a happy and harmonious society. This study has certain practical significance for further improving the leadership and management system of mental health education in schools, improving the level of mental health education of all teachers, promoting scientific research on mental health education among teachers, and improving the organization and implementation of mental health education in junior high schools.

## 3. Analysis of Mental Health Education Management Theories

Mental health is a relative concept and a continuous, positive, and efficient psychological state, which can have occasional disorders of behavior or minor mental disorders but can recover quickly through self-regulation and keep oneself in a state of internal and external harmony, with the ability to keep one's life in this good condition for a long time.

Teachers' mental health standards are reflected in many aspects, which are basically expressed as intelligence, personality, adaptability, self-regulation ability, and enthusiasm for work and life. The specific performance is as follows: (1) can accept his professional role happily, with good self-awareness and sound personality; (2) have a stable, positive, and optimistic emotional state; (3) have good professional quality and a sense of professional belonging and mission. Teachers should love their jobs and love their students; (4) have cheerful personality and good interpersonal relationships.

The article "A Survey of Teachers' Status in Mental Health Education Management Based on Big Data Analysis" was retracted in 2023. Reasons: signs of a paper mill; suspected computer-generated content; unreliable results or conclusions; concerns about the data.

The concept of mental health education management in colleges and universities is derived from education management theory and higher education management theory; that is to say, mental health education management in colleges and universities is based on the theory of education and management, supported by the technology of psychology, from the perspective of students' mental health, and fully coordinates various favorable conditions such as human, material, and financial resources within the school to efficiently carry out the mental health education in colleges and universities [13]. The goal and task of management are to make use of various resources of the school, coordinate various departments, establish the management system of college mental health education, conduct relevant questionnaires and psychological tests for students, then make a corresponding psychological assessment, establish students' mental health files, and formulate corresponding intervention or treatment plans, to effectively manage students' mental health and achieve the improvement of students' mental adjustment ability and psychological quality. The contents of the management mainly include related psychological knowledge propaganda, psychological activities, psychological testing, questionnaire survey, psychological crisis intervention, and follow-up work.

Educational management is divided into educational administration, which is the government's management of education according to the law, and school management, which is the school's management of its education. Therefore, to fully understand this, the concept must be based on relevant theoretical studies. Management activity is one of the earliest activities that emerged in human society, and people have different understandings of management. Management is such an activity where it performs certain functions to efficiently acquire, distribute, and use human efforts and material resources to achieve certain goals. Management is planning and maintaining a work environment for people working in a collective that enables them to accomplish their intended goals and tasks. Management is the achievement of a goal with the least amount of time, money, materials, or exertion. From the above definition, management includes the elements of collectivity, resources, efficiency, and goals.

Educational management is the management activities that people perform in the field of education. Thus, the definition of management is also applicable to educational management, but there are some differences compared to other management activities. Education is a kind of nurturing activity, and it is difficult to define a unified criterion in many aspects, such as the purpose of education, attitude toward learning, and the development of emotional values [14]. In terms of content, educational management includes the management of educational undertakings, the management of schools and other organizations, and the self-management of educational administrators. Therefore, we can refer to the understanding of other management activities when understanding educational management, but it is important to fully understand the differences. The so-called educational management is a series of activities that organize and coordinate the control of the educational system and is divided into educational administration and school management.

The article "A Survey of Teachers' Status in Mental Health Education Management Based on Big Data Analysis" was retracted in 2023. Reasons: signs of a paper mill; suspected computer-generated content; unreliable results or conclusions; concerns about the data.

The theory states that a business is a system that organizes various elements that are interconnected to achieve the set goals of the organization or its members. It and the surrounding environment interact dynamically with each other and, based on internal and external information feedback, and constantly complete self-adjustment to meet the needs between itself and the environment, as shown in Figure 1.

System management theory emphasizes the concept of system management to carry out organizational management, integrating materials, funds, personnel, and other resources that are not directly related to each other into a system, and all basic functions should function around the system management objectives.

The theory is applied to the management of secondary school mental health education; that is, the management of secondary school mental health education as a whole is regarded as a multilevel complete ecosystem, and the organizational structure, rules and regulations, team building, hardware configuration, financial guarantee, educational curriculum, practical activities, school culture construction, classroom atmosphere, interpersonal relationships among classmates, and school campus environment are all key parts of the system, as well as family relationships and social relationships. Family relationships, social relationships, etc. are also external to the system [15]. The theory requires that firstly, school administrators should take a holistic view and focus on the top-level design when doing mental health education planning; secondly, they should focus on the hierarchy of the internal structure. Because secondary school mental health education requires the participation of multiple subjects within the school, these subjects can be divided into different elements and different levels. In the management of mental health education, different elements and levels must be arranged in a coordinated manner so that all elements can cooperate. Again, there is openness inside and outside the system. Mental health education management in secondary schools has shown increasingly important characteristics under the current situation [16]. At the same time, students' mental health education requires family and society to cooperate with school work and play the educational cooperation, and the external environment of school management has a nonnegligible influence on it. Finally, there is the dynamic equilibrium of the development and stability of secondary school mental health education management. The system of secondary school mental health education, like all complex systems, has the inherent law of dynamic balance. As the subject of education, young people themselves are characterized by constant growth and change, and their internal and external environments are in a balance of development and stability. Therefore, the management of mental health education in secondary schools requires that the whole process of students' growth and success be carried out, with emphasis on coherence and progressiveness.

The article "A Survey of Teachers' Status in Mental Health Education Management Based on Big Data Analysis" was retracted in 2023. Reasons: signs of a paper mill; suspected computer-generated content; unreliable results or conclusions; concerns about the data.

## 4. Teacher Status Survey Design

According to the current problems in the incentive mechanism of education, questionnaires, interviews, and case studies were conducted to understand the causes of teachers' occupational stress and its influencing factors and their real views on the incentive issue and to analyze the general and intrinsic needs of teachers. 140 teachers participated in the questionnaire, including 51 males and 89 females; their ages ranged from 30 to 50 years old; 56 had a bachelor's degree, 70 had a secondary school degree, and 4 had a college degree; 27 had less than 5 years of teaching experience, 29 had 5-10 years of teaching experience, 70 had 10-20 years of teaching experience, and 14 had more than 20 years of teaching experience. There were 7 questions in this questionnaire, 4 single-choice, 1 multiple-choice, and 2 open-ended questions. In interpersonal communication and communication, people with mental illness can easily cause interpersonal tension at work, which affects the improvement of work efficiency; in the family, it is also very easy to produce various family conflicts; if mental illness is not timely dredged for them and if it develops to a serious level, it will also pose a threat to the safety of the family and society.

Educational administrators, teachers, and students in eight middle schools were selected for individual interviews and questionnaires for this study. The question types of the teacher questionnaire and student questionnaire included single-choice, multiple-choice, and open-ended questions. The student survey questionnaire consisted of single-choice and multiple-choice questions. The single-choice questions are basic information about the survey subject, the mental health education teachers in their schools, mental health education materials, and other basic information [17]. The multiple-choice questions are used to investigate the contents and forms of activities of school mental health education, the ways for students to obtain mental health education knowledge, and whether school mental health education improves students' mental health. The teacher survey questionnaire consists of three parts. The first part is the basic information on the survey subject such as gender, teaching age, title, professional academic degree, and teaching discipline. The second part of the survey mainly involved the six requirements for the organization and implementation of mental health education in the survey respondents' schools and a preliminary understanding of the organization and implementation of mental health education in the survey respondents' schools [18]. The third part is the teachers' evaluation of the organization and implementation of mental health education in schools.

The article "A Survey of Teachers' Status in Mental Health Education Management Based on Big Data Analysis" was retracted in 2023. Reasons: signs of a paper mill; suspected computer-generated content; unreliable results or conclusions; concerns about the data.

The purpose of the interview outline is to further understand the current situation of the organization and implementation of mental health education in junior high schools. The questions in the interview outline were designed to focus on the six requirements of the organization and implementation of mental health education in schools and to understand the relevant situations from the perspectives of school education administration, school administrators, and teachers, to provide reference materials for the improvement measures in the latter part of the dissertation. The author used the interview method, questionnaire method, and fieldwork to understand the current situation of the organization and implementation of mental health education in junior high schools in Yueyang city, as shown in Table 1.

The author has done a lot of preparatory work in the process of conducting school field surveys. First, the purpose and significance of the survey are clarified, and the survey plan and the survey respondents are selected. Then, appointments were made with relevant personnel for individual interviews and questionnaires. Next, interview the research subjects as scheduled, distributing teacher questionnaires and student questionnaires. Finally, the questionnaires were collected, the data were analyzed, and the outline of the interview was compiled. In this survey, 400 teachers' questionnaires were distributed, 372 valid questionnaires were returned, and the efficiency rate of teachers' questionnaires was 93%. The survey was mainly based on teachers' questionnaires, and students' questionnaires were used to help understand the situation of mental health education in schools. The author interviewed 33 people, including 3 leaders of education administration, 6 school administrators, 12 teachers (including 6 teachers of mental health education), and 12 students. The results of the questionnaire survey data statistics were illustrated using percentages, and the interview transcripts were used as a supplement to the questionnaire survey results. The field survey of this study was conducted on October 25, 2020, and this questionnaire survey was distributed and collected on-site.

The article "A Survey of Teachers' Status in Mental Health Education Management Based on Big Data Analysis" was retracted in 2023. Reasons: signs of a paper mill; suspected computer-generated content; unreliable results or conclusions; concerns about the data.

School administrators have effectively built the basic system of mental health education and made the useful exploration of the joint model of mental health education; the education administration attaches importance to training course directors and mental health education teachers, and the leading role of psychological head teachers in mental health education training has been brought into play [19]. Schools attach importance to the inculcation of teachers' mental health by the campus psychological environment, and school administrators pay attention to teachers' mental health status. Schools have established student mental health education files, richer mental health education materials, and more ways for students to obtain mental health knowledge, etc.

In terms of subject type differences, science students scored significantly higher than arts and physical education students in terms of intelligence, indicating that science students are more intelligent, are good at abstract thinking, have stronger learning ability, and have quicker and more correct thinking; in terms of emotional stability and persistence, arts and physical education students scored significantly higher than arts and physical education students, indicating that arts and physical education students are more emotionally stable and mature, able to face reality. Students of arts and sports scored significantly higher than students of science and arts and sports, indicating that students of arts and sports are more fantasy-loving, wild, unrestrained, self-reliant, and decisive but also slightly more skeptical, headstrong, and stubborn.

The analysis of the sample characteristics of the questionnaire revealed that 44 samples of mental health education demonstration schools, 107 samples of mental health education nondemonstration schools, and 52 samples were not clear about the classification of schools. Therefore, these “unclear” samples either belonged to nonmodel schools of mental health education or were teachers in model schools who did not care much about the management of mental health education in schools.

The article "A Survey of Teachers' Status in Mental Health Education Management Based on Big Data Analysis" was retracted in 2023. Reasons: signs of a paper mill; suspected computer-generated content; unreliable results or conclusions; concerns about the data.

## 5. Educational Management Strategy Design and Analysis

Today, when education is rapidly being conquered and integrated by the Internet, junior high school teachers must quickly learn to use the Internet to be competent in teaching, so that they will continue to study after their busy work, otherwise they will not be able to keep up with the times. Aiming at the current situation that junior high school teachers are under too much pressure in the survey, as the main body of pressure, teachers themselves must learn to adjust themselves, and the management should also take corresponding countermeasures in terms of teacher management, and the two sides should work together to relieve the pressure of junior high school teachers to the greatest extent. Teachers should change their ideas and release pressure scientifically. The government and schools should jointly build multiple platforms to enhance teachers' self-efficacy. Teachers should also strengthen respect and understanding for students and parents and at the same time improve their professional quality.

First, the highest score in the construction of mental health education publicity facilities indicated that teachers in the three schools thought that the schools did not do enough to promote and educate about mental health education; second, the high score in teachers' awareness of and attention to mental health and counseling indicated that teachers' awareness of these two aspects was insufficient; third, the lowest score in the implementation degree of psychological counseling indicates that teachers in the schools think that the schools are doing a better job in carrying out psychological counseling activities; fourth, the higher score in the self-assessment of teachers' mental health level indicates that teachers have a low evaluation of their mental health level; fifth, the lower score in the mental health education management system indicates that the schools have strengthened their attention to the management system aspect of mental health education.

A mental health education work team has been formed with members at all levels with a clear division of labor and responsibilities to implement individual counseling and developmental counseling. The two psychology teachers are full-time and part-time, each graduated in psychology and education, and have both psychology teacher qualification and psychological certification, which not only can serve the school's mental health education work at the practical level but also have achieved several awards and honors at the research level. Science students are more intelligent in comparison, are good at abstract thinking, have strong learning ability, and have quick and correct thinking.

The article "A Survey of Teachers' Status in Mental Health Education Management Based on Big Data Analysis" was retracted in 2023. Reasons: signs of a paper mill; suspected computer-generated content; unreliable results or conclusions; concerns about the data.

The most visible difference in teaching evaluation is the title. Title promotion can meet teachers' spiritual needs because it is a reflection of one's teaching and research ability; at the same time, title promotion can also meet teachers' material needs because it is linked to salary. However, title promotion is not something that can be decided by a certain unit or a certain person, and there are certain quotas for title evaluation every year, and there are many unethical practices in the process of title evaluation: serious seniority ranking, fake papers, watery work performance, etc. There are also many rigid indexes, especially about some certificates. To get the title as soon as possible, teachers must spend a lot of effort and make every effort to prepare for these certificates [20]. For example, if they want to give a lecture, they must give it in school first and then go to the district to give it after the school has passed it, and they must fight for the target; the district must win the first or second prize before they are qualified to give it in the city. This created a great deal of tension for teachers, as shown in Figure 2.

From outside the school, the higher education administrative department, as the superior agency directly guiding the implementation of the policy of general secondary schools in Shandong Province, should set up a special administrative department targeting the work of mental health education in the mental health education management system. It is mainly responsible for formulating local policies on mental health education, organizing training for teachers of mental health education in schools at all levels, allocating funds for mental health education work, and unifying the equipment of indoor facilities for psychological counseling, etc. It should be noted that because of the different scales of school operation and teaching levels, there should be different degrees of difference in the allocation of relevant mental health education resources to avoid the problem of uneven mental health education work. At the same time, it is necessary to set up a mental health education academic research department, which is mainly responsible for conducting in-depth research to keep the theory of mental health education up-to-date with the actual situation in the province, to provide the theoretical basis for the formulation of relevant policies [21]. It is also responsible for leading the mental health education teaching activities in general secondary schools in Shandong Province: through liaising with social mental health education groups to conduct mental health education awareness lectures for teachers and students in general secondary schools in the province, guiding subject teaching and psychology teacher training, etc.

The article "A Survey of Teachers' Status in Mental Health Education Management Based on Big Data Analysis" was retracted in 2023. Reasons: signs of a paper mill; suspected computer-generated content; unreliable results or conclusions; concerns about the data.

In other words, for the higher education administration department and its exclusive mental health education research institution, the staffing should be precise and complete, with Level 2 counselors and experts in psychology and education as the core strength, supplemented by relevant administrative staff. Mental health education teachers and counselors in school counseling rooms should have at least a bachelor's degree or higher in psychology, as well as one to three years of internship experience and a minimum qualification of counselor III [22]. According to the actual situation, a psychological counselor with psychological education training can be provided as an assistant to improve the teaching level and counseling effect as much as possible. Today's children's parents have “baby” with them, and the only child is loved by the whole family, and they are not under any pressure. That is why, when it is getting harder and harder for teachers, they feel more pressure and agree that this is the main source of anxiety in their work and life.

In addition to the traditional lecture method, classroom teaching can also be carried out through role-playing and situational drama to make students empathize and empathize, thus improving the efficiency of classroom teaching and enriching the content and form of teaching. The activities of quality development can enhance students' sense of teamwork, eliminate the gap between people, build a strong will, and organize students to attend various mental health education seminars to enrich their knowledge of mental health.

## 6. Analysis of Results

### 6.1. Analysis of the Results of the Research on the Status of Teachers

The questionnaire consists of two parts; the first part is the basic information of the participants, including four items, such as gender, education category, grade, major category, and family economic status. The second part is the content of the questionnaire, including self-assessment and other assessments of college student's mental health status, college students' views on the need for mental health education, and the status of existing mental health education [1].

There were significant differences among teachers of different age groups; there were also significant differences among teachers with different working years, and all of them showed a trend of decreasing mental health status with increasing age or working years, as shown in Figure 3. Teachers' mental health status gradually decreases with age and years of experience, which is also consistent with the findings of studies related to teachers as a group with a high prevalence of burnout. The age stages were divided into 20-30 years, 30-40 years, 40-50 years, and 50-60 years, and the working years were divided into less than 5 years, 5-10 years, 10-15 years, 15-20 years, and more than 20 years. Teachers of different ages and years of experience face different problems, and the older they are and the longer they have been in the profession, the lower their level of mental health, regardless of age group or years of experience, in relative terms.

The article "A Survey of Teachers' Status in Mental Health Education Management Based on Big Data Analysis" was retracted in 2023. Reasons: signs of a paper mill; suspected computer-generated content; unreliable results or conclusions; concerns about the data.

According to the analysis, young teachers who are younger and have relatively short working years show a higher level of mental health. Since new young teachers have just entered the workplace, they are not yet familiar with their jobs and specific job requirements and are in the stage of individual-environmental adaptation; thus, they have less work stress and have not yet developed obvious psychological problems [23]. At the same time, young teachers have simple family relationships, and in addition to work stress, they also have less life stress. Therefore, the mental health level of young teachers who are younger and have relatively shorter working years is generally higher.

Teachers in their 30s-50s and with 5-20 years of work experience showed a relatively good level of mental health. Middle-aged teachers in their 30s and 50s with 5 to 20 years of experience face not only physical and mental stress at work but also some stress from their family environment. Teachers at this age usually have families, and the cost of education for their children and support for their parents is increasing every year, so they are under high stress in terms of economic pressure and therefore have certain mental health problems [24].

With the development of the social economy, changing external environment, and rich campus life, students' demands on school mental health education management have become higher and more diversified, the professionalism of mental health education practitioners have become more demanding, and the inherent traditional education and management modes have failed to meet students' psychological needs, as shown in Figure 4. According to the survey results, the demand for mental health educators' professional background shows that the percentages of “psychology major,” “education major,” and “medicine” are 80.76%, 7.69%, 15.38%, and 7.69%, with “psychology” and “medicine” accounting for the highest percentages.

The article "A Survey of Teachers' Status in Mental Health Education Management Based on Big Data Analysis" was retracted in 2023. Reasons: signs of a paper mill; suspected computer-generated content; unreliable results or conclusions; concerns about the data.

From the above survey results combined with the structure of school teachers, it is easy to find that students have a strong demand for mental health teachers with professional backgrounds, there is a serious lack of resources for school mental health education management, and there is a serious lack of professional psychological teachers, with many nonprofessional counselors and class teachers acting as psychological teachers. Fully mobilize the enthusiasm of all school educators for mental health education services.

Although education administrators have a deeper and more comprehensive understanding of mental health education with the development of the times, in today's increasingly stressful employment situation, education management staff pay more attention to vocational training to achieve a good employment rate [25]. This makes mental health education “marginalized” in college education and simply fulfills the requirements of higher authorities. However, education administrators do not realize that the lack of continuous psychological treatment and crisis intervention makes the preliminary census work meaningless, and the complex and changing social environment may turn students' psychological problems into psychological crises at any time.

However, along with the development of society, teachers are facing great pressure and the incidence of psychological disorders is extremely high. Therefore, it is important to pay attention to not only the mental health of education but also the mental health of teachers. To increase the organizational culture, through different forms of training, effectively improve teachers' educational ability, and provide a platform for teachers to highlight and form a positive working atmosphere.

### 6.2. Educational Management Strategy Results

Different working environments have different effects on teachers. In the new era of education development, cultural environment building has become an important part of modern campus spiritual motivation. Practice shows that the cohesiveness of teachers is stronger in schools with a good culture. When the cultural atmosphere of the garden and the values of teachers are unified and when the campus culture fully reflects the respect for teachers, teachers will become one with the school, teachers will feel proud of their unit and willing to dedicate their wisdom to the garden, and this is where the power of campus culture is [26]. The school is not only a place to impart scientific and cultural knowledge but also a garden for sowing civilized and healthy thoughts and noble moral sentiments to the new generation. With the construction of civilized and healthy campus culture, we promote the great development of educational reform and teaching management and strive to cultivate a practical school characteristic with a cultural atmosphere. The face-to-face communication and communication between people have been reduced, making the human touch gradually weakened. Due to the lack of emotional support, people are prone to excessive pressure at work. With the increase of pressure, mental illnesses also appear with the development of the times and a gradual spreading trends.

The article "A Survey of Teachers' Status in Mental Health Education Management Based on Big Data Analysis" was retracted in 2023. Reasons: signs of a paper mill; suspected computer-generated content; unreliable results or conclusions; concerns about the data.

The mental health education program should be carried out in the richest possible form, and the work should emphasize not only the acquisition of knowledge but also the overall development of students' personalities and personalities, the acquisition of psychological skills, and learning to see problems from a psychological perspective. At the same time, enrichment activities suitable for different types and characteristics of students should be carried out based on in-depth and dynamic research of students' needs combined with the characteristics and laws of the subject. For example, according to the survey, 24.64% of students need online psychological counseling, but currently, the school does not provide this type of service.

In management, based on the summary of successes and failures, we should be good at exploring its strengths and gradually form a management style, methods, and teaching characteristics with our characteristics, and through the development of the individual characteristics of our school, we will be unique among our sister schools. We will cultivate team spirit, bring into play the group effect of relying on teachers to run the school, and build good campus culture [27].

Mental health education teachers work part-time in Civics or other disciplines. Since the head of the teaching and research group of Civics or other disciplines does not have a professional background in psychology, he or she may not be able to direct the work of mental health education. The number of working hours and salary of mental health education teachers are related to the professional development of the teaching and research group of Civics and Political Science subjects. This management model is not conducive to carrying out the organization and implementation of mental health education, as shown in Table 2.

In primary and secondary schools, students usually form their own outlook on life, values, and personality qualities, and the mental health of teachers is considered to be one of the key factors affecting their healthy growth. The questionnaire also revealed that about 75% of the teachers had received training related to mental health education during their current school work, and the frequency and level of training were high. However, the questionnaires and interviews revealed that many teachers still consider themselves to be deficient in their ability to educate students about mental health and have high expectations for the improvement of mental health education expertise and the ability to identify students' psychological problems. The reason for this is still that the training has not worked to achieve the expected effect.

The article "A Survey of Teachers' Status in Mental Health Education Management Based on Big Data Analysis" was retracted in 2023. Reasons: signs of a paper mill; suspected computer-generated content; unreliable results or conclusions; concerns about the data.

We divide the training here into two categories depending on the target audience. One type of training is for psychology teachers. Because the number of psychology teachers in each school is small, this type of training is mainly organized by the region or the psychology teachers themselves go out for training. The other type of training is for all teachers. Schools mainly organize this type of training themselves which is one of the reasons for the gap between nonmodel and model schools. First, mental health education is a very practical and hands-on job, but the current training format still mainly lectures, with less practical training, and the training is not systematic and continuous enough. It seems to be lively on the surface, but the actual effect is limited. Second, the number of psychological trainings for general teachers is low. Through interviews, we learned that most nonmodel schools provide psychology-related training for nonpsychology teachers about once or twice a semester, and many teachers believe that the frequency and content of such training do not address their confusion.

Looking at today, the pressure of education is increasing day by day, and the working environment of teachers is not very optimistic. Teachers will inevitably have various psychological problems. Schools must attach great importance to teachers' mental health. Therefore, to avoid the negative impact of the mental health of primary and secondary school teachers, the corresponding education management departments should change their thinking and not only pay attention to the mental health of students but also pay attention to the mental health of teachers.

## 7. Conclusion

Through questionnaires and in-depth interviews, this study constructed an evaluation index system that can reflect the actual situation of teachers' mental health levels based on the reference of previous evaluation indexes about teachers' mental health levels. The system mainly includes five primary indicators: positive attitude toward people, ability to understand things objectively, respect for students, understanding of parents, and professionalism, and 17 secondary indicators such as failure handling attitude, aggressiveness, and listening to parents' ideas. A more complete index system for evaluating the mental health level of primary and secondary school teachers can provide an effective reference and reference for improving the mental health level of primary and secondary school teachers. This study initially achieved the expected goal and suggested management suggestions for teachers' mental health from the education management and society levels, respectively, which meet the actual situation. For the education administration, it should regularly assess teachers' mental health levels, establish teachers' mental health records, reform teachers' work evaluation system, and provide teachers with mental health education; the society level should continue to improve teachers' external environment, create an atmosphere of respect for teachers, and improve teachers' living standard. The ideal goal of mental health education in colleges and universities is the scientific construction of a management system construction, promoting the effective implementation of various tasks, and helping college students understand mental health knowledge, optimize their psychological quality, enhance their psychological adjustment ability, and prevent and alleviate psychological-related problems through a series of mental health education courses and activities promptly. Although this research has achieved certain results, due to the limited time and energy, the number of research objects is not large enough. In the future, the number of research objects in this field can be increased to obtain more accurate conclusions.

The article "A Survey of Teachers' Status in Mental Health Education Management Based on Big Data Analysis" was retracted in 2023. Reasons: signs of a paper mill; suspected computer-generated content; unreliable results or conclusions; concerns about the data.

## Figures and Tables

**Figure 1:** System management theory model diagram.

**Figure 2:** Education management strategy.

**Figure 3:** Comparison of teachers' mental health status with different working years.

**Figure 4:** Professional background needs of students expected mental health workers.

**Table 1:** Basic information of teachers in the selected schools.

Title	Number of faculty and staff on board	Number of mental health education	Percentage
School A	168	1	0.60%
School B	105	2	1.90%
School C	253	3	1.19%
School D	224	2	0.89%
School E	145	1	0.69%
School F	168	2	1.19%
School G	135	1	0.74%
School H	289	3	1.04%

**Table 2:** Suggestions for improving the management of mental health education.

Options	Subtotal	Percentage
Individual counseling	752	17.37%
Group counseling	563	13.00%
Mental health courses	751	17.34%
Psychological testing	845	19.52%
Mental health seminar	597	13.79%
Online counseling	312	7.21%
Psychological club activities	479	11.06%
No benefit	31	0.72%
Total	4330	100.00%

## Data Availability

The data used to support the findings of this study are available from the corresponding author upon request.
